The article "Effects of Nonelastic Taping and Dual Task on Kinematics and Kinetics of the Ankle Joint" was published in 2021. Journal: J Healthc Eng.

# Effects of Nonelastic Taping and Dual Task on Kinematics and Kinetics of the Ankle Joint

**DOI:** 10.1155/2021/8866453

**Published:** 2021-02-28

**Authors:** TaoLi Wang, RongZhou Zhong, ShaSha Liu, GuoJiong Hu, WenXin Niu, YuBin Wang

**Affiliations:** ^1^Shanghai Yangzhi Rehabilitation Hospital, Shanghai Sunshine Rehabilitation Center, Tongji University School of Medicine, Shanghai 201615, China; ^2^Laboratory of Rehabilitation Engineering and Biomechanics, Tongji University School of Medicine, Shanghai 200092, China

## Abstract

**Objectives:**

The purpose of this experimental study was to investigate the effects of nonelastic taping and dual task on ankle kinematics and kinetics in gait analysis of healthy adults.

**Methods:**

A total of 21 healthy adults completed trials of gait analysis using a Vicon system combining ground walking with different cognitive task conditions (none, modified Stroop color/character naming, and serial-7 subtraction), with or without nonelastic taping. Ankle kinematics and kinetics including speed, ankle plantarflexion and inversion angle, ground reaction force (GRF), and stride time variability (STV) under all conditions of taping (YES or NO) and cognitive task (none, naming, and subtraction) were characterized and analyzed with repeated-measures ANOVA.

**Results:**

As regards cognitive performance, the serial-7 subtraction performance under walking conditions with and without taping was significantly poorer than simple sitting condition (*P* < 0.001). For kinematics and kinetics, STV showed statistically significant decrease (*P*=0.02) when subjects underwent taping application. Vertical GRF was significantly greater under taping than barefoot (*P*=0.001). Ankle plantarflexion at initial contact (IC) under the dual-task walking was significantly more than under simple walking (*P*=0.008).

**Conclusions:**

Applications of nonelastic taping and dual task may lead to the STV, vertical GRF, ankle plantarflexion, and speed alterations because of restricted joint range of motion and changed sensorimotor neural circuit. When healthy adults performed dual-task walking, central neural resources allocation was disturbed, leading to weakened performance in both motor and cognitive tasks.

## 1. Introduction

Ankle is one of the most vulnerable body sites in sports injuries and accounts for 10–30% of all sports injuries [1]; previous injuries could increase risk of reinjury by 88% [2]. Ankle sprain accounts for 80% or even more of ankle injuries [3].

Previous studies have suggested that feedforward mechanisms may also change in patients with ankle injuries [4–6]. Feedforward is a preprogrammed mechanism adopted by the central nervous system in motor control to deal with external disturbances, so as to obtain better motor control and equilibrium stability. The positioning of the ankle before landing during walking could be considered as one of the manifestations of a feedforward mechanism [7].

Moreover, central processing requires a certain degree of attention to acquire and integrate information and to further ignore unrelated stimuli during locomotion [8]. The central system handling two tasks simultaneously may activate motor control-associated areas in the brain, thereby leading to dual-task costs [4]. Like other daily activities, even simple walking requires the support of the central nervous system, as it needs high coordination of the body and motor control system activities with complete attention and cognitive ability [9]. A dual-task paradigm, where participants perform a cognitive task while walking, is typically used to investigate the relationship between cognition and gait performance [9]. Gait impairment during dual-task paradigm is thought to indicate interference or costs of competition between shared resources involved in both cognitive and gait tasks [9–11]. A systematic review showed that the overall effects of dual task on gait include decreased speed, decreased cadence, decreased stride length, increased stride time, and increased stride time variability [10].

Taping is widely used as a preventative and therapeutic intervention in sports rehabilitation, and it has been shown to decrease the risk of spraining the ankle again [12–14]. The mechanism of this reduction of risk is still unclear, although ankle taping may have an effect on restricting joint range of motion [15, 16], increasing mechanical stability [17], or working as a psychological reminder so as to consciously moderate lower limb-loading behavior [14]. Neither tape nor the strength of tape/skin interface alone could resist the force required to rupture lateral ankle ligament complex, but, when combined with the body tissues, taping would improve the capacity to dissipate the energy along with potentially traumatic forces [18]. It is recommended that future research address the effects of combining taping with rehabilitation or dynamic exercise [14, 19]. Kuni et al. [20] found that nonelastic taping stabilized the midfoot by reducing midfoot movements and rearfoot excursion in the frontal plane during drop landing in the healthy and those with chronic ankle instability.

Walking is one of the most functional activities of human and injuries often occur at initial contact during walking, especially when some external disturbance happens. Effects of nonelastic taping and cognitive tasks on gait performance of healthy adults could help to investigate the central mechanism of ankle injury and/or reinjury. Therefore, we hypothesized that the gait performance of healthy adults would be different under dual-task condition and be altered after the application of nonelastic taping on ankle. The purpose of the present study was to conduct an experiment to support it.

## 2. Methods

### 2.1. Research Design

This experimental study was designed to investigate effects of nonelastic taping and dual task on ankle kinematics and kinetics in gait analysis of healthy adults.

### 2.2. Participants

From January 2019 to September 2019, 21 healthy adults were recruited in Shanghai city as subjects. Exclusion criteria were as follows: (i) lower limb surgery, (ii) acute lower limb musculoskeletal injury in the previous three months, affecting joint integrity and function (sprains, fractures, etc.), (iii) any complaint about ankles in general (“giving way”, pain, instability, etc.), (iv) any abnormal alignment of lower limb joint due to diseases or traumas, and (v) accompanied by vestibular diseases, neurological conditions, and color blindness.

All subjects were tested for dominant leg. It was determined individually by asking which leg they would use to kick a ball as far as possible [21]. Subjects were informed of the objective of this experiment and signed an informed consent. This study was approved by the Medical Ethics Committee of the authors' institution (approval number: YZ2019-029).

### 2.3. Procedures

#### 2.3.1. Equipment

A three-dimensional motion capture system with eight Vicon MX T40-S cameras (Vicon Motion Systems Ltd., UK) was used for recording the kinematic data of the subjects' legs and feet. Data were recorded at 100 Hz using Vicon Nexus (1.8.5 vision) motion capture software. Three AMTI OR6 series force plates (Advanced Mechanical Technology Inc., USA) were used to record kinetic data at an acquisition frequency of 1,000 Hz.

#### 2.3.2. Taping

The rigid taping (Endura-FIX, China) was used in this study. The taping method applied in this study was commonly used [22]. All taping applications were performed by two senior therapists in our group. Two strips of taping were used for each tested ankle of subjects as planned. As shown in Figure 1, the taping started at the medial malleolus, passing through the sole of the foot, and stopped at the middle and lower third of the shank.

#### 2.3.3. Dual Task

In addition to ground walking at self-selected speed as motor task, cognitive tasks of the dual-task design were color/character naming (modified Stroop paradigm) [23] and serial subtractions of 7 [24], respectively. The former was to recognize the color of native language words while walking. The meaning of the words did not match the color. The subjects were asked to read the words silently to themselves and speak out the color verbally. The latter was consecutive subtractions by 7 while walking. For repeated subtractions by 7, a starting number was randomly selected from 200 to 250 (excluding those ending with 0 and 7). The subjects were asked to subtract 7 continuously from their minds and to speak out the results verbally.

#### 2.3.4. Markers Localization

The procedure of experiment was based on the working framework recommended by the International Society of Biomechanics [25]. A total of 23 infrared reflectors were localized: (i) pelvis (*n* = 5): anterior superior iliac spine, posterior superior iliac spine, and the spinous process of the second sacrum, (ii) hip joint (*n* = 2): the greater trochanter of the femur, (iii) knee joint (*n* = 6): lateral condyle of the femur, medial condyle of the femur, and the middle and lower 1/3 of the line connecting the greater trochanter to the lateral femoral condyle, (iv) ankle joint (*n* = 8): medial and lateral malleolus, the middle and lower 1/3 of the line connecting the fibula capitulum to lateral malleolus, and termination of the Achilles tendon, and (v) the second metatarsal head (*n* = 2). Operations in all the tests were performed by 2 designated therapists in our group.

#### 2.3.5. Data Acquisition

Before the experiment, the system and environment were calibrated. A 3s-long static calibration trial was collected with the participant in standing anatomic position to define anatomic neutral for the motions of interest. The subjects were given enough time to familiarize with the laboratory environment and explained with the main protocol of the testing process. All the subjects wore tight sports jackets and shorts for gait testing. The subjects with myopia wore their glasses. Firstly, the subjects were asked to walk two rounds in the established gait testing route to adapt. The time required to finish walking was recorded using a stopwatch.

Under bare feet and nonelastic taping application, each participant was subjected to gait testing under normal walking, color/character naming while walking, and serial-7 subtraction while walking in a counter balanced order. Each gait testing was repeated three times and average kinematic and kinetic data were collected for further analysis. The interval between each task condition was 120 s, and that between each walking test was 30 s. During the experiment, walking and cognitive tasks could not be interrupted, and instructions were given to avoid prioritization of either task. Walking could not be stopped even there were errors in the tasks. In addition, participants sat and completed as many color/character naming tasks and subtractions as possible within the same time, which was needed to complete the walking distance over the trial.

The total number of dual-task attempts and the number of correct answers in each testing by subjects in different task condition were recorded. To assess the serial-7 subtraction dual-task performance, a normalized response index was calculated based on Hayman's work (number of correct responses/number of total responses × 14) [26].

The selected indexes included walking speed, ankle dorsiflexion or plantar flexion and inversion angle at IC, maximal plantar flexion and inversion from 100 ms before IC to 80 ms after IC, ground reaction force (GRF) on the supporting foot in vertical, anterior to posterior (AP), and medial-lateral (ML) direction, and stride time variability (STV). The collected data were preliminarily processed in Vicon Nexus, and C3D files were obtained. Then, C3D files were input into Visual3D software (V5, C-Motion, USA) to further calculate the characteristic values of the required indicators. All GRF data were normalized based on body weight (BW).

### 2.4. Statistical Analysis

To determine the relevance of the results, 2-way repeated-measures (RM) ANOVAs were performed to analyze gait data of cognitive tasks under two walking conditions (barefoot and taping). Friedman's ANOVAs were used to determine the effect of cognitive task and taping application on cognitive task performance due to the data being nonparametric. Descriptive statistics were expressed by $\bar{X}$ ± *S*. *P* < 0.05 was considered as statistically significant. 95% Confidence Interval (CI) values for population means were based on *t*-distribution and equation (1) and were calculated as follows:

(1) $$\begin{array}{c} 95\%\text{CI}=\bar{X}\pm t_{\alpha /2,v}\frac{S}{\sqrt{n}}, \end{array}$$

where $\bar{X}$ is the mean value, *t* indicates *t*-distribution, *α* stands for type I error, *v* is degree of freedom, *S* is the standard deviation, and *n* is the sample size. All analyses were performed within SPSS 24.0 (IBM Corp., Armonk, NY, USA).

## 3. Results

### 3.1. Subject Characteristics

Twenty-one participants, 15 males and 6 females, completed the testing. The participants' mean age was 36.4 ± 10.8 years, mean height was 171.1 ± 8.4 cm, mean weight was 69.0 ± 8.3 kg, and mean BMI was 23.52 ± 2.09 kg/m^2^.

### 3.2. Cognitive Task Performance

Performance in the cognitive task is summarized in Table 1. Friedman's test and following Dunn-Bonferroni test revealed significant effects of walking on serial subtraction performance (*P* < 0.001) and only significant difference of correct number of character naming tasks under barefoot walking compared with sitting (*P*=0.02). The serial-7 performance of barefoot and taping walking was poorer than sitting condition.

### 3.3. Kinematics and Kinetics

Table 2 details the kinematic and kinetic data including speed, STV, ankle plantar flexion and inversion angle at IC, maximal plantar flexion and inversion from 100 ms before IC to 80 ms after IC, and vertical, anterior to posterior (AP), and medial-lateral (ML) components of GRF. Additionally, 95% Confidence Intervals for population means are shown in Table 3. Inversion is positive and plantar flexion is negative unless otherwise noted.

The gait speed was significantly slower under the dual-task condition compared to single walking task based on RM ANOVA tests (*F* = 9.007, *P*=0.003). There were no significant effects of taping on speed data (*F* = 4.283, *P*=0.053). There was no interaction effect between taping and cognitive task on speed *(F* = 0.331, *P*=0.721).

There was a main significant effect of walking conditions on STV, indicating that taping usage can avoid the instability induced by dual task (*F* = 6.506, *P*=0.020). The data of STV were lower under taping walking than under barefoot walking. There was no statistical significance of cognitive tasks on STV (*F* = 2.371, *P*=0.130). Although interaction between taping and cognitive tasks showed no significant effect, there was some tendency of STV under the influence of taping and cognitive task (*F* = 3.375, *P*=0.069) (Figure 2).

Plantar flexion at IC under the dual-task walking was significantly more than that under simple walking (*F* = 5.48, *P*=0.008). No statistical significance was found in plantar flexion at IC under the effects of taping (*F* = 1.302, *P*=0.269) and interaction between taping and cognitive task (*F* = 1.470, *P*=0.243). There were no statistical significances of maximal plantar flexion from 100 ms before IC to 80 ms after IC under taping (*F* = 3.997, *P*=0.061), cognitive task (*F* = 2.378, *P*=0.107), and their interaction (*F* = 1.008, *P*=0.375). In terms of ankle inversion at IC and maximal inversion from 100 ms before IC to 80 ms after IC, there were no significant effects under taping (*F* = 0.017, *P*=0.899; *F* = 0.882, *P*=0.36), cognitive task (*F* = 1.703, *P*=0.197; *F* = 0.479, *P*=0.623), and their interaction (*F* = 0.067, *P*=0.935; *F* = 0.607, *P*=0.55), respectively.

Time-normalized ankle angles of one typical participant in sagittal plane and frontal plane are shown in Figures 3 and 4. We observed a trend toward an increase in ankle dorsiflexion and inversion under dual-task condition and this tendency was restored after taping usage; however, no significant differences were noted.

There were significant effects of taping (*F* = 16.231, *P*=0.001) and interaction between taping and cognitive task (*F* = 4.87, *P*=0.013) on vertical component of GRF. Vertical GRF was significantly greater under taping walking than under barefoot walking. No significant difference was found in cognitive task on vertical GRF (*F* = 2.383, *P*=0.107). We found no significant effects under taping (*F* = 1.112, *P*=0.306; *F* = 2.066, *P*=0.168), cognitive task (*F* = 2.93, *P*=0.066; *F* = 0.802, *P*=0.456), and their interaction (*F* = 1.071, *P*=0.353; *F* = 2.217, *P*=0.124) on AP and ML GRF, respectively.

## 4. Discussion

Walking speed can be used as an indicator to reflect the overall functional status of human beings [27]. The walking speed of healthy people under dual task is lower than that under single task [10]. The results of speed data of the present study were in line with the previous research, which indicated that performing cognitive tasks during walking occupied central neural system resources linked to gait and then impaired the gait performance [10]. No significant effects of taping were found on speed; however, there was a restoring trend of speed after taping application. These results might be attributed to the fact that more proprioception input or other effects by nonelastic or rigid taping attracted participants' attention from cognitive task to motor task or just to working memory effect. When young people exercise, if their tasks and environment change, gait tends to produce more stable and less variable adaptive mechanisms [24]. When subjects with functional ankle instability performed dual-task walking, the ankle joint functioned around more supinated position [28]. Plantar flexion, inversion, and adduction occur in case of foot supination. At this time, the midfoot is locked and stiffness increases, while the stability of ankle joint could be reduced in the frontal plane.

Our study found significantly more ankle plantar flexion at IC under the dual-task walking, which matched previous studies [24, 28]. This could be due to a compensation to external disturbance (cognitive load) which made more stable midfoot or less variable movements. There were some anomalous values of ankle inversion, such as a small mean and large standard deviation. A major reason for this could be the fact that some participants presented inverted calcaneus (positive), while others showed everted calcaneus (negative) at IC. In addition, the behavior of rear foot during walking condition could be correlated with rear foot posture in staticity [29]. So other parameters might be needed to analyze ankle movements in the frontal plane in gait, such as specific movements variability in an appropriate form [28, 30].

In terms of GRF, significant effects were found in GRF vertical data under the taping and interaction between taping and cognitive task. Vertical GRF became greater after application of taping. One way to interpret this result was that usage of taping could enhance awareness or attention of ankle joint during walking and then lead to some alteration in sensorimotor processing.

The available evidence does support the application of taping for reducing the risk of spraining the ankle again [13]. However, a meta-analysis showed no positive effects of taping on proprioception in functional ankle instability despite the limitation of differences in participants studied, the type of taping used, the way in which the tape was applied, and the way proprioception was measured [12]. More recently, Tsikopoulos et al. [19] found no significant effects of any tape on dynamic balance in patients with chronic ankle instability based on the Star Excursion Balance Test only. Based on the above lines of evidence, it was plausible that the protective effect of tape for preventing ankle reinjury was not likely to be due to enhanced proprioception. There are several techniques of ankle joint taping [12, 19]. The taping method we used in this study had been frequently used clinically [22]. After taping application, the gait speed showed a restoring change under dual-task conditions, while gait speed became slower in dual-task walking than in simple walking. Moreover, STV during taping walking presented a significantly decreasing change compared to barefoot walking under dual task. The mechanism for these results might involve effects that ankle rigid taping restricted joint range of motion [12] and altered the sensorimotor neural circuit through focus of attention [31, 32]. Existing researches showed that external attention focus could be beneficial for the transfer of learning, acquisition, and retention of a postural control task following an ankle injury [31, 32].

Dual-task conditions could increase STV of gait [10]. Movement variability is inherent in all human movements [33]. Appropriate movements variability, a chaotic structure, is necessary for daily activities and sports, which can help to adapt with individual goals and environmental condition [30, 33]. However, too high movements variability (a random structure) had been connected with acute and chronic musculoskeletal injuries during locomotion, while too low variability (a periodic structure) could lead to rigid movements and poor capacity of adapting to the environments and tasks [33, 34]. Gait and other movements variability can reflect central neural motor control and provide an additional dimension of movement analysis besides standard means, maximum, minimum, and so on [33]. Previous studies showed conflicting results about effects of cognitive load on gait variability in young adults [35–40]. Some studies reported increased variability during dual task [35, 36] and several demonstrated decreased variability with dual-task [37, 38], while others showed no effects of dual task on gait variability [39, 40]. The present study showed significantly lower gait STV when subjects performed walking with nonelastic taping. Furthermore, STV showed an increasing trend conducting a cognitive task with barefoot walking, while the changing tendency became flatter after the application of taping. It could mean that dual-task condition might change the allocation of central neural resources and weaken the motor control. Additionally, taping usage could improve neuromuscular control and redirect high-level processing resources away from cognitive task toward the motor task.

Walking itself and walking speed both require activation of the frontal lobe of the brain and connection with the higher-level central neural networks. Therefore, when walking, a cognitive task will share the central neural networks, causing interference; then performance of one or both tasks could be decreased [4]. In existing literature, cognitive tasks were classified into 5 general domains according to their requirement and the mental processes needed to execute them [10]. The five task domains are reaction time, discrimination and decision-making, mental tracking, working memory, and verbal fluency tasks. Overall, cognitive tasks involving internal interfering factors seem to disturb gait performance more than those concerning external interfering factors. In the present study, the serial-7 performance under barefoot walking and taping walking was poorer than sitting, while character naming performance was not. One interpretation of these findings was that serial-7 task required more central neural network resources shared with walking task compared to character naming task.

Previously, some authors have proposed “posture first” paradigm; that is, young and healthy adults will give priority to posture tasks when facing both posture and cognitive tasks, unless they receive external instructions [41]. In the context of walking, it claims that healthy subjects spontaneously prioritize gait stability over success on the “secondary” cognitive task when no instructions are given about task prioritization [41]. However, experiments show that this is not always the case. Yogev-Seligrated et al. [42] proposed a new task priority and integration model. The unconscious strategy of dual-task priority in life involves primary factors including functional posture reserve, self-awareness-based hazard estimation and secondary factors about personal characteristics, such as personality, emotion, and professional background. Posture reserve includes muscle strength, core stability, flexibility, feedback, feedforward, sensory integration, adaptability, and higher-level cortical control. The interaction between posture reserve and hazard estimation affects the prioritization strategy of dual task. Complete postural reserve enables people to give more attention to cognitive tasks even when the risk of instability is high. Moreover, those with poor quality of hazard estimation still pay more attention to cognitive tasks when their postural reserve is insufficient, resulting in an increased risk of postural instability, subsequent falling, or injuries [42].

Researchers also suggested, based on the Yerkes–Dodson law, a U-shaped relation between cognitive demand and postural sway under dual-task conditions according to cognitive task complexity [43]. Furthermore, Ghai et al. [44] proposed that reinvolvement of higher motor centers during speech production in a dual task could cause central interference, which might impact the person's dual task and motor performance. So, they called for nonverbal dual tasks and/or more functional tasks being applied in the future research and rehabilitation regimes [44]. In the present study, the cognitive task and motor performance were both weakened. The results could indicate that cognitive resources were interfered and reallocated to motor task and cognitive task with a certain weight. It was consistent with the integrated model of task prioritization proposed by Yogev-Seligrated et al. [42]: task prioritization during walking involves the weighting of the motor and cognitive state during the specific dual-task situation, the functional reserve, and compensatory capabilities of both modalities.

The present study supported our hypothesis as mentioned in Introduction. Gait speed was decreased when subjects performed dual-task walking, and after usage of nonelastic taping there was a restoring trend. STV data showed a significantly decreasing change after taping usage and had an increasing tendency under dual-task walking which became flatter after taping application. Nonelastic taping and dual-task condition had interaction effects on vertical GRF.

This study also has several limitations. The complexity and representativeness of cognitive and motor tasks are still insufficient. More challenging tasks can be used as interference in the future. This study used only self-control and controlled clinical research including specific patient population as intervention group could be conducted in the future. Nonelastic taping was one kind of external supports, and the effects of the trials were specific according to taping type and method.

## 5. Conclusion

When healthy adults performed dual-task walking, the performance of both motor and cognitive tasks would be weakened due to disturbance of central neural resources allocation. Applications of nonelastic taping and dual task may lead to the STV, vertical GRF, ankle plantar flexion, and speed alterations. The mechanisms might involve the effects that ankle taping had on restricting joint range of motion, giving some external stimulus, and altering the sensorimotor neural circuit through attention focus. In the future, more functional and diversified cognitive tasks as well as more appropriate indicators such as movement variability should be applied in gait or other movements analysis with and without influence by external supports to get more information on sensorimotor control in populations.

## Figures and Tables

**Figure 1:** Nonelastic taping application. (a) Lateral view. (b) Medial view.

**Figure 2:** Stride time variability (STV) during different task conditions.

**Figure 3:** Ankle joint dorsiflexion/plantar flexion. Dorsiflexion is positive. 0 = initial contact. Different color represents corresponding cognitive and walking status.

**Figure 4:** Ankle joint inversion/eversion. Inversion is positive. 0 = initial contact. Different color represents corresponding cognitive and walking status.

**Table 1:** Cognitive task performance.

	Sitting	Barefoot walking	Taping walking
Character naming			
Attempts (*n*)	9.24 ± 0.62	8.95 ± 0.67	9.33 ± 0.80
95% CI	(8.95, 9.52)	(8.65, 9.26)	(8.97, 9.70)
Correct (*n*)	9.19 ± 0.68	8.38 ± 0.74*∗*	8.95 ± 0.86
95% CI	(8.88, 9.50)	(8.04, 8.72)	(8.56, 9.35)
Error (*n*)	0.05 ± 0.22	0.57 ± 0.93	0.38 ± 0.59
95% CI	(−0.05, 0.15)	(0.15, 0.99)	(0.11, 0.65)
Accuracy rate (%)	99.47 ± 2.42	94.00 ± 9.52	96.01 ± 6.31
95% CI	(98.37, 100.57)	(89.66, 98.33)	(77.07, 91.19)

Serial-7 subtraction			
Attempts (*n*)	9.05 ± 0.59	8.10 ± 1.00*∗*	8.57 ± 0.81
95% CI	(8.78, 9.32)	(7.64, 8.55)	(8.20, 8.94)
Correct (*n*)	8.86 ± 0.73	6.38 ± 1.86*∗∗*	7.24 ± 1.55*∗*
95% CI	(8.53, 9.19)	(5.54, 7.23)	(6.53, 7.94)
Error (*n*)	0.19 ± 0.40	1.71 ± 1.35*∗∗*	1.33 ± 1.24*∗*
95% CI	(0.01, 0.37)	(1.10, 2.33)	(0.77, 1.90)
Response index	13.70 ± 0.63	10.86 ± 2.80*∗∗*	11.78 ± 2.17*∗*
95% CI	(13.42, 13.99)	(9.59, 12.14)	(10.79, 12.76)

Compared with sitting, *∗*significance with *P* < 0.05 and *∗∗*significance with *P* < 0.001.

**Table 2:** Kinematics and kinetics of barefoot walking and taping walking under different task conditions.

	Barefoot			Taping			*p* value		
	None	Naming	Subtraction	None	Naming	Subtraction	Cognitive	Walking condition	Interaction effect
Speed (m/s)	1.24 ± 0.10	1.23 ± 0.08	1.14 ± 0.13	1.27 ± 0.06	1.28 ± 0.11	1.17 ± 0.17	0.003^*∗*^	0.053	0.721
STV (%)	4.55 ± 4.34	5.94 ± 4.37	6.80 ± 4.83	3.79 ± 2.77	3.59 ± 2.90	3.98 ± 2.49	0.130	0.020^*∗*^	0.069
Plantar flexion (IC) (°)	−5.15 ± 3.30	−6.97 ± 3.30	−5.83 ± 1.99	−4.64 ± 3.14	−5.58 ± 2.61	−5.63 ± 3.01	0.008^*∗*^	0.269	0.243
Inversion (IC) (°)	−0.53 ± 5.70	0.23 ± 6.09	0.13 ± 5.99	−1.21 ± 5.35	0.29 ± 4.51	0.26 ± 5.18	0.197	0.899	0.935
Maximal plantar flexion (°)	−10.79 ± 2.78	−12.00 ± 2.62	−11.96 ± 2.57	−10.23 ± 3.15	−10.57 ± 3.15	−11.32 ± 3.93	0.107	0.061	0.375
Maximal inversion (°)	1.91 ± 4.65	1.83 ± 4.67	1.96 ± 3.90	0.04 ± 5.59	0.77 ± 4.82	0.67 ± 5.91	0.623	0.360	0.550
Vertical GRF (N kg^−1^)	0.89 ± 0.12	0.86 ± 0.12	0.81 ± 0.13	0.90 ± 0.10	0.97 ± 0.14	0.90 ± 0.16	0.107	0.001^*∗*^	0.013^*∗*^
AP GRF (N kg^−1^)	0.19 ± 0.03	0.19 ± 0.05	0.17 ± 0.02	0.18 ± 0.03	0.20 ± 0.04	0.18 ± 0.03	0.066	0.306	0.353
ML GRF (N kg^−1^)	0.01 ± 0.02	0.02 ± 0.02	0.02 ± 0.02	0.02 ± 0.04	0.01 ± 0.02	0.03 ± 0.03	0.456	0.168	0.124

*∗*Significant differences with *P* < 0.05. AP, anterior-posterior; GRF, ground reaction force; IC, initial contact; ML, medial-lateral; STV, stride time variability.

**Table 3:** 95% confidence intervals for means.

	Barefoot			Taping		
	None	Naming	Subtraction	None	Naming	Subtraction
Speed (m/s)	1.24 (1.19, 1.28)	1.23 (1.19, 1.27)	1.14 (1.08, 1.2)	1.27 (1.24, 1.3)	1.28 (1.23, 1.33)	1.17 (1.09, 1.25)
STV (%)	4.55 (2.46, 6.65)	5.94 (3.83, 8.05)	6.80 (4.47, 9.12)	3.79 (2.45, 5.12)	3.59 (2.2, 4.99)	3.98 (2.78, 5.18)
Plantar flexion (IC) (°)	−5.15 (−6.74, −3.56)	−6.97 (−8.56, −5.39)	−5.83 (−6.79, −4.87)	−4.64 (−6.15, −3.13)	−5.58 (−6.84, −4.32)	−5.63 (−7.08, −4.18)
Inversion (IC) (°)	−0.53 (−3.28, 2.21)	0.23 (−2.71, 3.16)	0.13 (−2.76, 3.02)	−1.21 (−2.79, 2.37)	0.29 (−1.88, 2.46)	0.26 (−2.24, 2.76)
Maximal plantar flexion (°)	−10.79 (−12.13, −9.45)	−12.00 (−13.27, −10.74)	−11.96 (−13.2, −10.72)	−10.23 (−11.75, −8.71)	−10.57 (−12.09, −9.05)	−11.32 (−13.21, −9.42)
Maximal inversion (°)	1.91 (−0.33, 4.15)	1.83 (−0.42, 4.08)	1.96 (0.08, 3.84)	0.04 (−2.66, 2.74)	0.77 (−1.55, 3.1)	0.67 (−2.17, 3.52)
Vertical GRF (N kg^−1^)	0.89 (0.83, 0.94)	0.86 (0.8, 0.92)	0.81 (0.75, 0.87)	0.90 (0.85, 0.95)	0.97 (0.9, 1.04)	0.90 (0.82, 0.98)
AP GRF (N kg^−1^)	0.19 (0.18, 0.2)	0.19 (0.17, 0.21)	0.17 (0.16, 0.18)	0.18 (0.17, 0.2)	0.20 (0.18, 0.22)	0.18 (0.16, 0.19)
ML GRF (N kg^−1^)	0.01 (0, 0.02)	0.02 (0.01, 0.03)	0.02 (0.01, 0.02)	0.02 (0.01, 0.04)	0.01 (0, 0.02)	0.03 (0.01, 0.04)

## Data Availability

All data are available upon request to the corresponding author Wenxin Niu via e-mail (niu@tongji.edu.cn).
